# Low Iron Diet Increases Susceptibility to Noise-Induced Hearing Loss in Young Rats

This article has been retracted.

**DOI:** 10.3390/nu8080456

**Published:** 2016-07-28

**Authors:** Fei Yu, Shuai Hao, Bo Yang, Yue Zhao, Jun Yang

**Affiliations:** 1 Department of Nutrition and Food Hygiene, School of Public Health, China Medical University, No. 77 Puhe Road, Shenyang North New Area, Shenyang 110122, China; ford_cmu@163.com (Y.Z.); yangjun@mail.cmu.edu.cn (J.Y.); 2 Department of Otolaryngology, First Affiliated Hospital of China Medical University, No. 155, Nanjing North Street, Heping District, Shenyang 110001, China; kellya@163.com (S.H.); feigo_dl@163.com (B.Y.)

**Keywords:** iron deficiency without anemia, ribbon synapse, spiral ganglion cell

## Abstract

We evaluated the role of iron deficiency (ID) without anemia on hearing function and cochlear pathophysiology of young rats before and after noise exposure. We used rats at developmental stages as an animal model to induce ID without anemia by dietary iron restriction. We have established this dietary restriction model in the rat that should enable us to study the effects of iron deficiency in the absence of severe anemia on hearing and ribbon synapses. Hearing function was measured on Postnatal Day (PND) 21 after induction of ID using auditory brainstem response (ABR). Then, the young rats were exposed to loud noise on PND 21. After noise exposure, hearing function was again measured. We observed the morphology of ribbon synapses, hair cells and spiral ganglion cells (SGCs), and assessed the expression of myosin VIIa, vesicular glutamate transporter 3 and prestin in the cochlea. ID without anemia did not elevate ABR threshold shifts, but reduced ABR wave I peak amplitude of young rats. At 70, 80, and 90 dB SPL, amplitudes of wave I (3.11 ± 0.96 µV, 3.52 ± 1.31 µV, and 4.37 ± 1.08 µV, respectively) in pups from the ID group were decreased compared to the control (5.92 ± 1.67 µV, 6.53 ± 1.70 µV, and 6.90 ± 1.76 µV, respectively) (*p* < 0.05). Moreover, ID without anemia did not impair the morphology hair cells and SGCs, but decreased the number of ribbon synapses. Before noise exposure, the mean number of ribbon synapses per inner hair cell (IHC) was significantly lower in the ID group (8.44 ± 1.21) compared to that seen in the control (13.08 ± 1.36) (*p* < 0.05). In addition, the numbers of ribbon synapses per IHC of young rats in the control (ID group) were 6.61 ± 1.59, 3.07 ± 0.83, 5.85 ± 1.63 and 12.25 ± 1.97 (3.75 ± 1.45, 2.03 ± 1.08, 3.81 ± 1.70 and 4.01 ± 1.65) at 1, 4, 7 and 14 days after noise exposure, respectively. Moreover, ABR thresholds at 4 and 8 kHz in young rats from the ID group were significantly elevated at 7 and 14 days after noise exposure compared to control (*p* < 0.05). The average number of young rat SGCs from the ID group were significantly decreased in the basal turn of the cochlea compared to the control (*p* < 0.05). Therefore, ID without anemia delayed the recovery from noise-induced hearing loss and ribbon synapses damage, increased SGCs loss, and upregulated prestin after noise exposure. Thus, the cochleae in rat pups with ID without anemia were potentially susceptible to loud noise exposure, and this deficit may be attributed to the reduction of ribbon synapses and SGCs.

## 1. Introduction

Iron deficiency (ID), the most common form of micronutrient deficiency, is the primary cause of anemia, which affects more than two billion people, especially children and pregnant women [1,2,3,4]. Although half of anemia cases are due to iron deficiency anemia (IDA), the most severe form of ID, the prevalence of ID without anemia, is three to five times greater than IDA [5]. Importantly, emerging studies support that ID without anemia during fetal brain development can have negative consequences on neurotransmission and myelination in the auditory pathway with auditory brainstem response (ABR) displaying abnormally decreased wave amplitudes and increased inter-wave latencies [6,7,8,9]. Currently, we only measure hematological data including hemoglobin (Hb), serum level of iron (SI), hematocrit (Hct) and serum ferritin (SF), which is not optimal for reflecting the iron status of the animals. However, to some extent, we might draw a conclusion that animals did not develop anemia by these hematological data. We only established a model of nonanemic maternal ID during pregnancy and lactation, and the offspring showed signs of ID, without signs of severe anemia.

Noise exposure is the common cause of hearing loss, which adversely affects the cochlea, auditory nerve and transmission of neural impulses [10]. Traditionally, the largest influence of noise exposure on the ear and hearing appears at early postexposure times. Although noise exposure at relatively low levels or intensities can induce temporary hearing threshold shifts, this kind of noise-induced acute injury to cochlea is reversible [11]. Recently, a nationwide cohort study in Sweden suggests that occupational noise exposure during pregnancy is associated with future hearing dysfunction in children [12]. It is thus imperative to elucidate the mechanisms of auditory dysfunction and the relationship between ID without anemia and noise exposure in the inner ear.

The coding of sound information relies on synaptic transmission being both reliable and temporally precise by the hair cell afferent synapse [13]. The cochlear ribbon synapses are the first afferent neuronal connection, and capable of accurate neurotransmitter release between inner hair cells (IHCs) and SGCs [14,15,16]. The ribbon synapses connect many synaptic vesicles by a pre-synaptic ribbon. A120 kDa protein is selectively enriched in ribbon fraction and is named RIBEYE, which is the major structural component of synaptic ribbon [17]. The domain B of RIBEYE includes a partial carboxy terminal binding protein 2 (CtBP2) sequence for staining patterns [18]. In addition, Myosin VIIa and vesicular glutamate transporters (VGLUT) 3 are two proteins that have important roles in vesicle function. Myosin VIIa contributes to regulate vesicle cycling of cochlear hair cells, and VGLUT3 contributes to the loading of glutamate into the synaptic vesicles [19,20]. Another protein, prestin, the outer hair cell (OHC) motor protein, contributes to OHC electromotility [21]. A recent study showed that mild maternal IDA downregulated VGLUT3 and myosin VIIa, and upregulated prestin in the cochleae of young guinea pigs [22]. Nevertheless, little is known regarding the involvement of myosin VIIa, VGLUT3 and prestin expression in the cochlea following ID without anemia and noise exposure. Consequently, the present study was designed to explore the effects of ID without anemia on the cochleae in young rats before and after noise exposure by physiological and morphological alterations. Therefore, we attempted to ascertain whether ID without anemia could primarily affect the inner ear of offspring by increasing its sensitivity to noise exposure. This hypothesis was tested by comparing the sensitivity to noise-induced hearing loss in normal rats versus ID rats in the absence of anemia.

## 2. Materials and Methods

### 2.1. Animals and Diets

Procedures involving laboratory animals were performed in accordance with the general principles of the Institutional Animal Care and Use Committee. All protocols were approved by China Medical University Institutional Animal Care and Use Committee with a protocol number of CMU62033008. Sprague-Dawley rats (200 ± 10 g) with a normal Preyer’s reflex, were obtained from the Center for Experimental Animals (National Animal Use License number: SCXK-LN2013-0007) of China Medical University. Animals were individually housed with free access to water and food in an established animal house with a controlled temperature of 22 ± 2 °C, a relative humidity of 55% ± 15%, and a 12-h light/dark cycle. These female rats were randomly assigned to one of two dietary groups as follows: One group (control group; *n* = 10) was fed a control diet (iron content: 103.95 ± 31.71 mg/kg diet, measured by atomic absorption spectrometry). The content of iron was prepared in the laboratory by adding ferrous sulfate heptahydrate instead of ferric citrate, to the formula for the AIN-93G purified rodent diet guidelines [23]. The other group (iron deficient group; *n* = 10) was fed an iron deficient diet (iron content: 25.27 ± 9.08 mg/kg diet). These ingredients were based on prior studies [24,25]. Table 1 showed the composition of experimental diets. After acclimation for 2 weeks, two female rats with one proven male rat were placed for mating at the same time. All female rats were examined the next day for presence of the vaginal plug. The day the vaginal plug was found was considered as Gestational Day (GD) 0. Each litter was culled to 10 pups on Postnatal Day (PND) 4, equating as much as possible the number and pups of each sex in a given litter. Offspring were weaned on PND 21, and transferred to plastic hanging cages (two per cage) until PND 36. A diet regimen began two weeks before mating and through the remainder of the experimental period. Throughout the study period, each animal, including the pups, was observed at least once daily for weight and any signs of morbidity, or toxicity. Hearing measurements were collected on each evaluation time point by ABR recording (eight ears per group) in this study. After animals were anesthetized, ABR audiograms were obtained on each evaluation time point. On PND 21, 12 animals per group were decapitated under deep anesthesia, and cochlear tissues were quickly removed from the skull and separated. On PND 36, seven animals per group were decapitated and cochlear tissues were collected. On PND 22, 26 and 29, four animals per group were decapitated and cochlear tissues were collected.

### 2.2. Iron Status

Measurements of iron status were performed as previously described [24,26]. Blood samples of dams (0.5 mL/per animal) were collected on GD 7, 14, and 21 by alternately clipping the toenails for serum level of iron (SI), hematocrit (Hct) and serum ferritin (SF) measured. Blood samples of dams were collected on PND 21 by direct cardiac puncture for hemoglobin (Hb), SI, Hct and SF measurements after deep anesthesia with ethyl ether. In addition, blood samples of pups were collected by clipping the toenails for Hb and SF measurement on PND 21, and were collected after ABR measurement by direct cardiac puncture for Hb and SF measurements on PND 36 (14 days after the noise exposure). After blood samples were collected, serum was separated (3000 rpm, 5 min) and stored at −70 °C. Serum samples were analysis for iron concentrations SI by atomic absorption spectrophotometry. Hb was measured by using a colorimetric cyanmehemoglobin method. Hct was measured by blood centrifugation in micro-capillary tubes and read in a microhematocrit reader. SF was measured by using Ferritin ELISA Kit and read in a microtiter plate reader. Hb and Hct Kits used were obtained from Nanjing Jiancheng Biotechnology (Jiancheng, Nanjing, China).

### 2.3. Hearing Measurements

Hearing function of offspring was measured by ABR testing as previously described [22]. Control and ID pups were sedated using 10% chloral hydrate (0.45 mL/kg, Sigma, St. Louis, MO, USA) and we examined an ABR recording in a soundproof chamber before exposure (on PND 21), following exposure on the 1st day (on PND 22), 4th day (on PND 26), 7th day (on PND 29) and 14th day (on PND 36) after noise exposure. ABRs were obtained with subcutaneous silverwire electrodes being inserted ventrolateral to the right ear (active) and at the vertex (negative) with a ground electrode inserted at the lower back. The sound delivery tube of an insert earphone was tightly fitted into the external auditory canal. A subcutaneous needle electrode active lead was positioned at the vertex and referred to the second electrode at the tip of the nose. The ground electrodes were located over the neck muscles. Tone burst stimuli, with a 0.2 ms rise/fall time (cosine gate) and 1-ms flat segment at frequencies of 4, 8, 16, and 32 kHz, were generated, and the amplitude was specified by a sound generator and attenuation real-time processor and programmable attenuator (Tucker-Davis Technology, Alachua, FL, USA). Sound-level calibrations were performed using a Sound Level Meter (Rion, Tokyo, Japan). ABR waveforms were recorded for 12.8 ms at a sampling rate of 40,000 Hz using 50- to 5000-Hz band-pass filter settings; waveforms from 256 stimuli at a frequency of 9 Hz were averaged. ABR waveforms were recorded in 10-dB sound pressure level (SPL) intervals down from a maximum amplitude until no waveform could be visualized. The ABR threshold was defined as the lowest intensity capable of eliciting a replicable, visually detectable response that displayed at least two peaks and a minimum amplitude of 0.5 µV. ABR wave I amplitude was analyzed following a previous method [27]. Each wave at high levels (70–90 dB SPL) is made up of one negative (n) deflection and one positive (p) deflection. This positive peak is followed by a negative deflection. ABR wave I amplitude analysis consists of three parts: time of peak (from beginning to Ip), SPL of click and amplitude of wave I (Ip-In) (latency, 1.2–1.9 ms). An algorithm for an automated determination of ABR amplitudes was programmed in MATLAB (MathWorks) [27].

### 2.4. Noise Exposure

Control and ID pups were exposed to noise on PND 21 following previous methods [10,27]. Animals were exposed in separate stainless steel wire cages, to white noise at 100 dB SPL for 2 h to induce temporary threshold shifts, in a ventilated sound-exposure chamber. The sound chamber was fitted with speakers (YH25-19B, 25 W, 16 Ω, Zhenmei Electronics, Tianjin, China) driven by a noise generator (33,220 A, Yachen Electronics, Dongguan, China) fed from noise software. The noise sound files were created and equalized with audio editing software (Audition 3; Adobe System, Inc., San Jose, CA, USA). Sound levels were calibrated with a sound level meter (model 1200; Quest Technologies, Oconomowoc, WI, USA) at multiple locations within the sound chamber to ensure uniformity of the sound field. Sound levels were measured before and after exposure to ensure stability.

### 2.5. Cochlear Tissue Processing and HE Staining

The cochleae of control and ID pups were removed on PND 21 and PND 36 following a previous method [28]. After ABR measurement under deep anesthesia, the temporal bone was then removed and the cochlea was quickly separated. The round and oval windows were opened, and they were perfused with 2.5% glutaraldehyde for scanning electron microscopy (SEM) or 4% paraformaldehyde for immunostaining at 4 °C overnight. The cochlea shell was separated from the basal turn under a dissecting microscope in 0.1 M phosphate-buffered saline (PBS, pH 7.2). The parietal gyrus of the basilar membrane was also separated. In addition, the vestibular membrane and cover membrane were removed. The auditory nerves were processed for light microscopy using the standard method consisting of fixation in formalin, decalcification using EDTA, embedding in celloidin, serial sectioning along the cochlear modiolus direction at a section thickness of 20 μm, and staining of every sixth section using hematoxylin–eosin (HE) staining. SGC counts were performed for the basal, middle, and apical turns of the cochleae on the HE-stained sections [10]. The areas of Rosenthal canal and the cochlear turn were quantified by measuring their cut surfaces using ImageJ software. All neurons meeting the size and shape criteria to be considered type 1 SGCs within each profile of Rosenthal canal were counted for the basal, middle, and apical turns of the cochleae. The SGC density was determined as the number of cell nuclei per 10,000 μm^2^ Rosenthal canal.

### 2.6. Electron Microscopy

The SEM was examined on PND 21 and PND 36 following a previous method [29]. The cochlea was perfused with 2.5% glutaraldehyde and fixed at 4 °C for 24 h. The organ of Corti was dissected using an anatomy microscope. The tissues were post-fixed with 1% osmium tetroxide in 0.1 M PBS for 2 h at room temperature and dehydrated in graded ethanol solutions from 50% to 100% (each for 30 min). Then, the specimens were dried in an HCP-2 critical point dryer, and sputter-coated with platinum for 4 min in an E-102 ion sputter. The specimens were examined by a JEOL JSM-35C SEM (Hitachi 7100, Tokyo, Japan). The images were recorded digitally and photographed. Cell density was defined as the number of counted cells from a distance along the basilar membrane, and divided by that distance. The average densities of IHCs and OHCs were calculated for each cochlea. The average cell counter per 100 μm were analyzed in the cochleae to obtain values of cell densities of IHCs and OHCs by using a log-linear model (Poisson regression) for Count with log (Distance) as an offset and a random effect for variation between preparations [30].

### 2.7. Immunofluorescence

On PND 21 and PND 36, the separated basilar membranes of control and ID pups were fixed in 4% paraformaldehyde and dissolved in 0.1 M PBS with 30% sucrose for 1 h at room temperature. Next, these samples were washed three times in 0.01 M PBS and preincubated for 30 min at room temperature in blocking solution of 5% normal goat serum in 0.01 M PBS with 0.3% Triton X-100, then were incubated with rabbit anti-CtBP2 (1:50, ABCam, Cambridge, UK), rabbit anti-myosin VIIa (1:200, Santa Cruz, CA, USA), rabbit anti-VGLUT3 (1:200, ABCam) or goat anti-prestin (1:200, Santa Cruz) left at 4 °C for 24 h. Then, the incubated samples were washed out in 0.01 M PBS for three times, and incubated with the secondary antibody Alexa Fluor 488 goat anti mouse IgG (1:200, Invitrogen, Carlsbad, CA, USA), Alexa Fluor 568 goat anti rabbit IgG (1:200, Invitrogen) or Alexa Fluor 488 donkey anti goat IgG (1:200, Invitrogen) at 37 °C for 2 h. After incubation, the samples were washed in PBS twice. After dropping a small amount of DAPI (4′, 6-diamidino-2-phenylindole; Santa Cruz, CA, USA) in the slide, basement membranes were tiled under a dissecting microscope; the coverslip covered the slide. The samples were imaged directly with a confocal laser scanning microscope (FV1000, Olympus; emission wavelengths 488 and 568 nm) to test the specificity of the primary antibody. The number of RIBEYE/CtBP2 positive spots was counted in each IHC. To determine the average number of labeled spots in each IHC, total values of labeled spots from 7 to 10 IHCs of per location (the basal, middle, or apical turn) in each cochlea (8 cochleae per group) were counted, and then the average numbers of labeled spots in each IHC were calculated.

### 2.8. Western Blotting

On PND 21 and PND 36, fresh cochlear tissue of control and ID pups were homogenized in 250 μL of buffered isotonic cocktail containing protease and phosphatase inhibitors. The protein concentrations of the supernatant were measured based on the Bradford method with bovine serum albumin as a standard. Tissue lysates were diluted to contain the same concentration of protein (3 μg/μL) and were boiled for 5 min. Next, 10 µL aliquots of each sample (containing 30 μg protein) were loaded onto 10% SDS-acrylamide gels. Proteins were separated by application of a constant voltage of 100 V for 90 min and then transferred onto nitrocellulose membranes at a constant voltage of 10 V for 45 min. After blocking the nonspecific sites with PBS containing 0.1% Tween 20 and 5% defatted dried milk, membranes were washed and incubated with primary antibody (rabbit anti-myosin VIIa, 1:500, Santa Cruz; rabbit anti-VGLUT3, 1:200, ABCam; goat anti-prestin, 1:500, Santa Cruz; rabbit anti-glyceraldehyde 3-phosphate dehydrogenase (GAPDH), 1:500, Santa Cruz) overnight at 4 °C and then incubated with horseradish peroxidase-conjugated secondary antibody (rabbit anti-goat, 1:500, Zhongshan Biotechnology, Beijing, China; goat anti-rabbit 1:500 dilution, Zhongshan Biotechnology). Blots were developed with the Easy Enhanced Chemiluminescence Western Blot Kit (Transgen Biotech, Beijing, China). Protein bands were subsequently quantified with an image analysis program (Gel Image System Ver. 4.00, Tianneng Technology, Shanghai, China).

### 2.9. Statistical Analysis

All data were expressed as mean ± SEM. SPSS for Windows, version 12.0, (SPSS Inc., Chicago, IL, USA) was used for statistical analysis. Student *t*-test and Chi square test were used to analyze the difference. The statistical significance was defined as *p* less than 0.05.

## 3. Results

### 3.1. ID without Anemia Leads to Growth and Iron Status of Young Rat Effects

The dams between two groups showed a similar number of successful parturitions, and similar weight gain, duration of gestation and feed intake (Table 2 and Table 3). The body weights of the pups increased steadily between the two groups throughout the observation period. There were no statistically significant differences in the SI and Hct in dams between control and ID group on GD 13 and 21 (*p* > 0.05). However, dams from ID group exhibited a significantly decreased level of SF on GD 13 and 21 compared to control (*p* < 0.05). On PND 21, there were no statistically significant differences in the Hb, SI and Hct in dams between the two groups (*p* > 0.05), but dams from the ID group exhibited significantly decreased level of SF compared to control (*p* < 0.05). In addition, there were no statistically significant differences in the Hb in pups between two groups on PND 21 and 36 (*p* > 0.05). However, pups from the ID group exhibited a significantly decreased level of SF on PND 21 and 36 compared to control (*p* < 0.05). Table 4 showed the number of preparations/cochleas used in different analyses performed.

### 3.2. ID without Anemia Reduces ABR Wave I Peak Amplitude of Young Rats

To evaluate peripheral and central auditory functions, we used ABR hearing thresholds in response to various stimuli. Figure 1A shows that ABR wave I amplitude analysis included amplitude of wave I, time of peak and SPL of click. Figure 1B shows the mean ABR thresholds between the control and ID group at varying tone pip frequencies (kHz). On PND 21, the average ABR thresholds of young rats from the ID group were not significantly different compared to the control at 4, 8, 16 and 32 kHz (Figure 1B, *p* > 0.05). Table 2 shows that the amplitudes of the wave I peak of young rats from the ID group were significantly decreased compared to control (*p* < 0.05), accompanied by hearing threshold elevation. In addition, the mean latency of the wave I peak of young rats from the ID group was not significantly different compared to the control (Table 5, *p* > 0.05).

### 3.3. ID without Anemia Lacks Significant Disruption in Hair Cells and SGCs Morphology of Young Rats

SEM shows the morphological changes of stereocilia and auditory nerve fibers in cochlear hair cells of young rats between the control and ID group (Figure 2A,B). There were no significant disruptions in the morphology and arrangement of the IHCs and OHCs of young rats from the ID group (Figure 2B). The stereocilia of IHCs and OHCs showed normal appearance between the two groups. HE staining shows the morphological changes of SGCs located in the cochlear postsynaptic region of young rats between the control and ID group (Figure 2C,D). There were no significant differences in the density of SGCs of young rats in the ID group compared to the control. DAPI staining shows the morphology and arrangement of the nuclei of cochlear hair cells of young rats between the control and ID group (Figure 2E,F). There were no significant disruptions in the morphology and arrangement of the nuclei of hair cells of young rats from the ID group.

### 3.4. ID without Anemia Delays the Recovery from Noise-Induced Hearing Loss in Young Rats

To evaluate the recovery of auditory functions, we tested ABR thresholds at frequencies of 4, 8, 16 and 32 kHz at 1, 4, 7 and 14 days after noise exposure for young rats between the control and ID group. Figure 3A,B shows that ABR thresholds at 4 and 8 kHz in young rats from the ID group were significantly elevated at 7 and 14 days after noise exposure, compared to the control (*p* < 0.05). That is, at 4 and 8 kHz, ABR thresholds in ID young rats after noise exposure showed a delayed recovery of temporary threshold shift components and a significant increase in permanent threshold shift. In addition, at 4 and 8 kHz, ABR thresholds in control young rats recovered to baseline (before noise exposure) from seven days after noise exposure. Figure 3C,D shows that ABR thresholds at 16 and 32 kHz in young rats from ID group also reflected a delayed recovery of temporary threshold shift compared to control, but these differences did not reach statistical significance (*p* > 0.05).

### 3.5. ID without Anemia Increases SGCs Loss in the Basal Turn of the Cochleae of Young Rats after Noise Exposure

HE staining was used for the quantitative changes in SGCs of the cochleae between the control and ID group before and after noise exposure. Figure 4A,B shows the representative sections of the basal turn of the cochleae between the control (Figure 4A) and ID group (Figure 4B). The average number of young rat SGCs from the ID group were significantly decreased in the basal turn of the cochleae compared to the control (*p* < 0.05). There were no significant differences in the density of SGCs of young rats from the ID group in the apical and middle turns of cochleae compared to the control (*p* > 0.05).

### 3.6. ID without Anemia Delays the Recovery from IHC Ribbon Synapses Damage in Young Rats after Noise Exposure

To estimate synaptic plasticity of IHC [16,29], immunostaining for RIBEYE/CtBP2 was used for the quantitative changes in ribbon-containing synapses per IHC between the control and ID group before and after noise exposure. We obtained acceptable recordings from 15 cells in each animal at each time point. Figure 5 showed that the majority of ribbon synapses were located inside the cochlear IHCs. Adjacent optical sections of the basal turn were used to count the number of ribbon synapses. Before noise exposure (on PND 21), the mean number of ribbon synapses per IHC was significantly lower in the ID group (8.44 ± 1.21) compared to that seen in the control (13.08 ± 1.36) (*p* < 0.05). In the control, the numbers of ribbon synapses per IHC of young rats were 13.08 ± 1.36 before noise exposure, and 6.61 ± 1.59, 3.07 ± 0.83, 5.85 ± 1.63 and 12.25 ± 1.97 at 1, 4, 7 and 14 days after noise exposure, respectively (Figure 5, panel of control). The number of ribbon synapses markedly decreased after noise exposure, with the maximal reduction occurring at four days after noise exposure compared with that seen before noise exposure (*p* < 0.01). The number of ribbon synapses was partially restored at seven days after noise exposure, although it was still less than before noise exposure (*p* < 0.05). The number of ribbon synapses was completely restored at 14 days after noise exposure. There was no significant difference in the number of ribbon synapses at 14 days after noise exposure compared with that seen before noise exposure (*p* > 0.05). In the ID group, the numbers of ribbon synapses per IHC were 8.44 ± 1.21 before noise exposure, and 3.75 ± 1.45, 2.03 ± 1.08, 3.81 ± 1.70 and 4.01 ± 1.65 at 1, 4, 7 and 14 days after noise exposure, respectively (Figure 5, panel of ID). Although the number of ribbon synapses was partially restored at 7 and 14 days after noise exposure, the number of ribbon synapses did not reach its status before noise exposure (*p* > 0.05).

### 3.7. ID without Anemia Does Not Regulate Myosin VIIa, VGLUT3 and Prestin in Young Rat Cochleae of before and after Noise Exposure, but Upregulates Prestin in the Cochleae after Noise Exposure

Myosin VIIa plays a pivotal role in vesicle cycling of cochlear hair cells, and VGLUT3 contributes to load glutamate into the synaptic vesicles [19,20]. Another protein, prestin, OHC motor protein, is necessary for OHC electromotility [21]. Myosin VIIa, VGLUT3 and prestin were expressed in young rat cochleae between two groups (Figure 6). Western blot revealed a single reactive band with an approximate molecular weight of 250 kDa, 65 kDa and 35 kDa, as anticipated. There were no significant differences between the control and ID group in myosin VIIa, VGLUT3 and prestin levels in young rat cochleae before and after noise exposure (*p* > 0.05). In the control, prestin was upregulated in the cochleae after noise exposure compared with that seen before noise exposure (*p* < 0.05). In the ID group, prestin was also upregulated in the cochleae after noise exposure (*p* < 0.05). In addition, at 14 days after noise exposure, a significant upregulation of prestin was observed in the cochleae of the ID group compared to the control (*p* < 0.05).

## 4. Discussion

We used a novel dietary restriction model to investigate the effect of ID in the absence of anemia on the cochleae of young rats before and after noise exposure. Interestingly, we observed no significant differences in ID-related ABR threshold changes and between the control and ID rats before noise exposure, we only observed a significant difference in the amplitudes of wave I peak between two groups. Thus, ID without anemia did not induce hearing impairment in young rats before noise exposure in our study. Most interestingly, we showed that recovery from noise-induced hearing and ribbon synapses injury was significantly impaired in this ID model in the absence of anemia, accompanied by the increase of SGCs loss and upregulation of prestin in the cochleae.

This rat model has also been used to induce ID without anemia by dietary iron restriction [24]. Recently, studies related to the models of limited iron availability have provided important viewpoint, but these models were often used to induce anemia, the most severe form of ID. Thus, in this study, our motivation was to observe the role of iron in ribbon synapses before and after noise exposure. To differentiate the different results between ID and IDA, we tested various ID diets on Sprague-Dawley rats and found a standard powdered rodent diet supplemented with ferric citrate (control: 0.735 g/kg diet including 123 mg iron, ID group: 0.315 g/kg diet including 53 mg iron). This model could represent a model of nonanemic maternal ID in which dams never developed anemia, ensuring that the growing embryos were not affected by hypoxia. Furthermore, the pups were still feed with the ID diet, and were not significantly anemic from birth to PND 36. However, the iron contents of the two diets in this study were relatively high. These ingredients were based on prior studies [24,25]. In these studies, the iron content of the control diet is 70–145 mg/kg diet, the iron content of the ID diet is 8.44–30 mg/kg diet. We acknowledge that the iron content of the control diet was variable (104 ± 32 mg/kg diet) and this amount of variability is not acceptable for a controlled feeding study. Although SI, Hct and SF of dams and pups were measured to reflect the model feasibility, the assay could not fully characterize the iron status of the animals. Furthermore, the measurement could not directly express the stability of the compounds. In fact, the test diets were a standard powdered rodent diet following the AIN-93G purified rodent diet guidelines [23] supplemented with ferric citrate. The ferric citrate was supplemented (control: 0.735 g/kg diet, ID group: 0.315 g/kg diet) and administered admixed with a powdered diet [24,25]. Thus, the content values were, in theory, 123 mg iron/kg feed in the control diet, and 53 mg iron/kg feed in the ID diet. To be able to ensure good handling by the animals, the components of the diets were thoroughly mixed and made into pellets. However, our pelletizing process affected the concentration of iron in the feed, especially regarding the stability of the iron content. This is because six samples of the control diet and ID die were analyzed, and iron content was detected at 103.95 ± 31.71 mg/kg feed and 25.27 ± 9.08 mg/kg feed, respectively. Moreover, this model showed that dams did not develop anemia while on the diet during pregnancy and lactation periods, ensuring that the growing embryos and infants were not affected by hypoxia. Moreover, the pups still received this kind of ID diet at weaning, and did not appear to have anemia. The pups born to the ID dams showed a decrease in iron storage capacity. We, therefore, think it reasonable to evaluate the potentiality of this experimental condition as the proposed model for this study. However, we did not measure transferrin saturation, transferrin receptor, total iron binding capacity, or tissue iron concentrations to fully characterize the iron status of the dams and pups. We understand that the iron status of the animals is imperative to reveal the role of iron during development on auditory nerves [31]. With regard to measurements of Hb, SI, Hct and SF, Hb is a late indicator of iron deficiency, SI is used to measure the amount of circulating iron that is bound to transferring, Hct reflects the volume percentage of red blood cells in blood, SF is an indicator of iron storage in vivo. Hb, SI, Hct and SF may not be optimal to reflect the iron status of the animals, but should be sufficient to draw a conclusion that animals did not develop anemia and reflect the model feasibility. Thus, ID group animals exhibited decreased SF and normal Hb, SI and Hct, which reflected decreased iron storage in vivo, and did not develop ID anemia.

Iron plays an important role in proper axonal maturation [31]. Iron supplement contributes to maintaining the integrity of the blood-labyrinth barrier and the homeostasis in the cochlea [32]. The main iron-related gene variants, such as *FPN1* (ferroportin), *TF* (transferrin), *HFE* (human hemochromatosis gene), and *HEPC*/*HAMP* (hepcidin), may be significantly associated with increased risk of developing sudden hearing loss [33]. Thus, the imbalance of iron homeostasis may impair inner ear anatomy and hearing.

The ABR recording is regarded as one of the auditory threshold measurements to observe auditory acuity, neural transmission times along the peripheral and brain stem portions of the auditory pathway [34]. Our study showed that ID without anemia could not elevate ABR thresholds (hearing loss), but could decline ABR wave I peak amplitudes of young rats before noise exposure, which reflected the summed activity of the remaining auditory nerve fibers. The elevated ABR threshold only reveals a general impairment in brain function [31]. The reduced ABR wave I peak amplitude indicates the impaired ribbon synapses between cochlear IHCs and type 1 SGCs [27]. To directly investigate the structural and functional relationship between ABR wave I peak amplitude and anatomy, we isolated the cochlear basilar membrane and observed the ribbon synapse density by immunofluorescence for RIBEYE/CtBP2, which is a prominent component of the synaptic ribbons anchored to the active zone of pre-synaptic specialization [35]. More importantly, cochlear ribbon synapse is the primary target of ototoxicity exposure, and is a sensitive nanostructure that can be easily affected by external factors [29]. As expected, ID without anemia caused the reduction of ribbon synapse density of young rats before noise exposure, but the ID offspring showed no disruption in the morphology of hair cells and SGCs. In addition, our analysis of myosin VIIa, VGLUT3 and prestin expression in the cochleae revealed no significant change in the expression of vesicle function related proteins and OHC protein before noise exposure. Thus, we postulated that ID-induced synaptic injury had not yet reached the status of hearing loss. This may be related to auditory function having a time-delay reaction to cochlear ribbon synapse under relatively mild injuries.

Our study further explored the idea that ID offspring in the absence of anemia could be potentially more susceptible to noise-induced hearing loss. Iron is important for brain development during fetal life and early childhood, as it supports neuronal and glial energy metabolism, neurotransmitter synthesis and myelination [36]. Although ID without anemia shows no disruption in myelin thickness or compaction, ID without anemia disrupts the normal development of the auditory nerve and results in altered conduction velocity in young rats [31]. The arrival of auditory nerve axons coincides with migration of most cochlear nucleus neurons. Furthermore, this interaction between auditory nerve axons and cochlear nucleus neurons is a critical part of proper brainstem development and synaptic maturation [37]. Following the loss of SGCs, the cell bodies of the auditory nerve fibers eventually match the loss of auditory nerve fiber synapses [38]. It seems likely that developmental ID without anemia could limit the recovery of synaptic connections and SGCs. On the other hand, noise exposure at low levels or intensities may induce temporary hearing threshold shifts, which could be related to the restoration of ribbon synapse [27]. That is, the reduction of ribbon synapse density is transient. Ribbon synapses may recover after this noise exposure [11]. These deficits may be attributed to impaired recovery from noise injury [10]. We therefore hypothesized that the morphological changes of ribbon synapses might induce impaired recovery from noise exposure in ID cochleae without anemia. In particular, ribbon synapses in the basal turn of the cochleae are more susceptible to ototoxic exposure [27]. We observed that ID without anemia impaired the recovery from noise-induced ribbon synapses injury in the cochlear IHCs of young rats, which corresponded with the changes of hearing thresholds after noise exposure. We therefore hypothesized that the other morphological changes observed in the cochleae might contribute to the elevated hearing thresholds in ID young rats after noise exposure. To test this hypothesis, we observed SGC density in the cochleae. As is well known, SGCs are the relay station for auditory information between hair cells and brain stem cells [39]. Furthermore, degeneration of SGCs is irreversible [27]. Although the present and previous studies did not observe the SGC loss after noise exposure at relatively mild stimulation [27], ID without anemia reduced the number of SGCs in the basal turn of the cochleae of young rats after noise exposure. We also observed that the SGC loss in the apical and middle turns of cochleae in ID young rats after noise exposure did not reach statistical significance. This may be due to the age of the animals, methods of dietary restriction and noise exposure [40]. Taken together, these suggested that the offspring with ID might be potential susceptible individuals to noise exposure.

The current study revealed the unexpected finding of no disruption in expression of myosin VIIa and VGLUT3 in the cochlear tissue of ID offspring after noise exposure. Myosin VIIa contributes to the endocytosis of IHCs, and VGLUT3 contributes to the glutamate transport of synaptic vesicles [19,20]. Thus, the present data indicated that ID without anemia could not disrupt endocytosis in IHCs and glutamate transport of synaptic vesicles in young rats after noise exposure, at least temporarily. Unlike myosin VIIa and VGLUT3, prestin, OHC motor protein, was upregulated in the cochleae of ID offspring after noise exposure. It is possible that upregulation of prestin could be part of a systems-level attempt to compensate for the hearing impairment, which may be a homeostatic mechanism [21]. In present study, the animals were examined in ABR test, which is a noninvasive neurophysiological assessment for auditory neural myelination. However, we did not perform DPOAE test, which is an ideal noninvasive assessment of the transduction sensitivity in OHCs, and may reflect losses and/or diminished function of a moderate number of OHCs. Thus, this could be one limitation of the current study, and further studies should be performed to develop the new normative data on the auditory system that would be of value to others.

## 5. Conclusions

In summary, low iron diet reduced the ribbon synapse density of young rats, and did not lead to hearing loss before noise exposure. However, the cochleae in rat pups with low iron diet were potentially susceptible to loud noise exposure, and this deficit may be attributed to the reduction of ribbon synapses and SGCs.

## Figures and Tables

**Figure 1:** Hearing test (auditory brainstem response (ABR) recording) on Postnatal Day (PND) 21 (before noise exposure). Representative illustration of the method to measure wave I of click (**A**); and threshold shifts of ABRs (**B**). Changes in the ABR threshold shift of young rats were not significantly different between the control (*n* = 8, right ear) and iron deficiency (ID) group (*n* = 8, right ear) at 4, 8, 16 and 32 kHz (*p* > 0.05).

**Figure 2:** Morphological analysis on PND 21 (before noise exposure). Representative scanning electron microscopy (SEM) images of young rat inner hair cells (IHCs) and outer hair cells (OHCs) in the control (*n* = 4, left ear, (**A**)) and ID group (*n* = 4, left ear, (**B**)), suggesting normal morphological characteristics of hair cells in the sensory epithelium. Scale bars = 20 µm. Representative HE staining of examination of young rat spiral ganglion cells (SGCs) in control (*n* = 4, right ear, (**C**)) and ID group (*n* = 4, right ear, (**D**)), showing unaffected morphology of postsynaptic SGCs in cochleae between two groups. Black arrows indicate SGCs. Scale bars = 50 µm. Representative confocal microscopy images reveal a normal morphological array of the young rat IHCs and OHCs in the control (*n* = 4, left ear, (**E**)) and ID group (*n* = 4, left ear, (**F**)), including one row of IHCs and three rows of OHCs. Blue labeling indicates DAPI-positive hair cell nuclei. Scale bars = 10 µm.

**Figure 3:** Hearing test (ABR recording) after noise exposure. ABR threshold shift of young rat between control (*n* = 8, right ear) and ID group (*n* = 8, right ear) at: 4 (**A**); 8 (**B**); 16 (**C**); and (**D**) 32 kHz before noise exposure (on PND 21) and 1, 4, 7 and 14 days after noise exposure. Data are mean ± SEM. * *p* < 0.05, as compared to control.

**Figure 4:** Quantitative changes in SGCs of the cochleae at 14 days after noise exposure (on PND 36). HE staining of changes in the number of young rat SGCs in control (*n* = 4, right ear, (**A**)) and ID group (*n* = 4, right ear, (**B**)). A large number of SGCs was present in the basal turn of the cochleae in the control (**A**); A decreased number of SGCs was present in the basal turn of the cochleae in the ID group (**B**); Black arrows indicate SGCs. Scale bar = 50 μm. Means of SGCs density of in the apical, middle, and basal turns of the cochleae were compared between groups (**C**). * *p* < 0.05, as compared to the control.

**Figure 5:** Quantitative changes of RIBEYE/CtBP2 in inner hair cell (IHC) ribbon synapses before and after noise exposure. Representative samples from the basal turn of the cochleae with each RIBEYE/CtBP2 punctum representing a synaptic ribbon. All immunostained synaptic ribbons are seen below the nuclei of IHCs (green) and between the IHCs and SGCs. IHC nuclei are stained using DAPI (blue). White arrows indicate ribbon synapses (green). Scale bar = 5 μm. Confocal microscopy of changes in the number of young rat synaptic ribbons between control (*n* = 4, left ear) and ID group (*n* = 4, left ear) at each evaluation time point. Before noise exposure (on PND 21), large numbers of ribbon synapses were present in young rat cochleae from the control (panel of control). The decreased number of ribbon synapses was present in young rat cochleae from the ID group (panel of ID). In addition, the number of ribbon synapses of the two groups decreased instantly at 1, 4, 7 days after noise exposure. Maximal reduction of ribbon synapses of two groups appeared at four days after noise exposure compared with that before noise exposure. The numbers of ribbon synapses of two groups increased at seven days after noise exposure compared with that at four days after noise exposure, but was still less than that before noise exposure. There was no significant difference in the number of ribbon synapses in the control between 14 days after noise exposure and before noise exposure. There was no significant difference in the number of ribbon synapses in the ID group between 14 days after noise exposure and 7 days after noise exposure.

**Figure 6:** Expression of myosin VIIa, vesicular glutamate transporter (VGLUT3) and prestin in the cochleae before noise exposure (on PND 21) and at 14 days after noise exposure (on PND 36). Representative immunoblots of myosin VIIa, VGLUT3 and prestin of young rat cochleae in control (left ear, *n* = 3) and ID group (left ear, *n* = 3) at respective time point (**A**); GAPDH was used as a loading control. Densitometry of immunoblots of myosin VIIa (**B**); VGLUT3 (**C**); and prestin (**D**) were compared, respectively, between two groups. The height of each bar represents the mean ± SEM (* *p* < 0.05).

**Table 1:** Composition of control and iron deficient rat diets.

Ingredients (g/kg Diet)	Control	ID
Cornstarch	529.5	529.92
Casein (>85% protein)	200.0	200.0
Sucrose	100.0	100.0
Soybean oil	70.0	70.0
Fiber	50.0	50.0
Mineral mix (Ferric citrate)	35.0 (0.735)	34.58 (0.315)
Vitamin mix	10.0	10.0
l-Cysteine	3.0	3.0
Choline bitartrate	2.5	2.5

**Table 2:** Reproductive and iron outcomes of dams and pups.

Group	Control	ID
Number of dams	10	10
Number of successful parturition	10	10
Duration of gestation (day) ^a^	21.0 ± 0.0	21.2 ± 0.5
Maternal weight gain (g) a GD 0–21	98.3 ± 18.3	96.9 ± 22.5
PND 4 sex ratio (male:female)	50:45	56:44
PND 4 body weights (g) ^a^	10.11 ± 2.22	8.61 ± 1.49
PND 7 body weights (g) ^a^	13.62 ± 2.12	12.21 ± 3.29
PND 14 body weights (g) ^a^	25.93 ± 3.34	23.36 ± 5.31
PND 21 body weights (g) ^a^	45.79 ± 1.43	43.11 ± 5.03
PND 28 body weights (g) ^a^	82.23 ± 10.16	79.77 ± 10.09
PND 35 body weights (g) ^a^	122.92 ± 12.79	112.85 ± 19.56
GD 13		
SI (µmol/L) ^a^	95.07 ± 18.81	90.50 ± 13.22
Hct	0.45 ± 0.13	0.44 ± 0.11
SF (mg/L) ^a^	5.19 ± 1.53	3.51 ± 1.07 *
GD 21		
SI (µmol/L) ^a^	97.38 ± 23.05	90.92 ± 20.34
Hct	0.46 ± 0.16	0.44 ± 0.19
SF (mg/L) ^a^	6.04 ± 1.61	3.98 ± 1.36 *
PND 21		
Dam		
Hb (g/L) ^a^	126.40 ± 17.62	115.08 ± 20.06
SI (µmol/L) ^a^	110.19 ± 29.03	96.90 ± 26.11
Hct	0.40 ± 0.17	0.39 ± 0.15
SF (mg/L) ^a^	6.29 ± 1.43	4.16 ± 1.19 *
PND 21		
Pups		
Hb (g/L) ^a^	117.46 ± 13.51	108.72 ± 13.79
SF (mg/L) ^a^	5.28 ± 1.33	3.61 ± 1.02 *
PND 36		
Pups		
Hb (g/L) ^a^	127.23 ± 20.06	114.07 ± 16.45
SF (mg/L) ^a^	5.53 ± 1.06	3.07 ± 1.10 *

GD, gestational day; Hb, hemoglobin; Hct, hematocrit; PND, postnatal day; SF, serum ferritin; SI, serum level of iron. ^a^ Mean ± SEM; * *p* < 0.05, compared to control.

**Table 3:** Feed intake ^a^ (g/day/animal) of control and iron deficient dams.

Group	Control	ID
GD 3	21.49 ± 3.96	22.12 ± 3.88
GD 6	26.74 ± 5.98	25.90 ± 4.45
GD 7	27.85 ± 7.04	25.52 ± 3.80
GD 9	30.74 ± 7.45	25.06 ± 4.11
GD 11	27.41 ± 5.65	25.42 ± 5.54
GD 14	29.30 ± 2.78	26.75 ± 3.91
GD 17	29.02 ± 3.97	29.76 ± 4.90
GD 20	22.59 ± 7.68	25.94 ± 6.95
PND 1	24.57 ± 7.29	23.48 ± 5.56
PND 4	34.95 ± 4.05	37.89 ± 7.89
PND 7	44.96 ± 6.00	46.21 ± 6.38
PND 14	63.75 ± 6.48	61.09 ± 7.68

GD, gestational day; PND, postnatal day. ^a^ Mean ± SEM.

**Table 4:** The number of preparations/cochleas (*n*) used in the different analysis performed of the pups.

Analysis Method	Control (32 Ears)	ID (32 Ears)
Hearing test ABR recording		
PND 21	8 (right ear)	8 (right ear)
PND 22	8 (right ear)	8 (right ear)
PND 26	8 (right ear)	8 (right ear)
PND 29	8 (right ear)	8 (right ear)
PND 36	8 (right ear)	8 (right ear)
Morphological test		
SEM (PND 21)	4 (left ear)	4 (left ear)
Immunofluorescence		
DAPI-positive nuclei (PND 21)	4 (left ear)	4 (left ear)
RIBEYE/CtBP2 (PND 21)	4 (left ear)	4 (left ear)
(PND 36)	4 (left ear)	4 (left ear)
HE staining (PND 21)	4 (right ear)	4 (right ear)
(PND 36)	4 (right ear)	4 (right ear)
Western blotting	3 (left ear)	3 (left ear)

ABR, auditory brainstem response; CtBP2, carboxy terminal binding protein 2; DAPI, 4′, 6-diamidino-2-phenylindole; GD, gestational day; HE staining, hematoxylin–eosin staining; PND, postnatal day; SEM, scanning electron microscopy.

**Table 5:** Amplitudes of wave I in pups’ clicks from 70 to 90 dB sound pressure level (SPL).

SPL (dB)	Control		ID	
	A of Wave Ip ^a^	Latency of Ip ^a^	A of Wave Ip ^a^	Latency of Ip ^a^
70	5.92 ± 1.67	1.49 ± 0.13	3.11 ± 0.96 *	1.56 ± 0.17
80	6.53 ± 1.70	1.35 ± 0.15	3.52 ± 1.31 *	1.44 ± 0.16
90	6.90 ± 1.76	1.29 ± 0.17	4.37 ± 1.08 *	1.35 ± 0.10

A, amplitude (µV); Latency of Ip, the latency of wave I (ms). ^a^ Mean ± SEM; * *p* < 0.05, compared to control.

## Abbreviations

The following abbreviations are used in this manuscript:

ABR	auditory brainstem response
CtBP2	carboxyterminal binding protein 2
DPOAE	distortion product otoacoustic emission
GAPDH	glyceraldehyde 3-phosphate dehydrogenase
GD	gestational day
Hb	hemoglobin
Hct	hematocrit
HE staining	hematoxylin–eosin staining
ID	iron deficiency
IDA	iron deficiency anemia
IHC	inner hair cell
OHC	outer hair cell
PND	postnatal day
SEM	scanning electron microscopy
SI	serum level of iron
SF	serum ferritin
SGC	spiral ganglion cell
SPL	sound pressure level
VGLUT	vesicular glutamate transporter
